The article "Research on the Current Situation, Causes, and Countermeasures of Primary School Physical Education Teachers' Health Literacy" was retracted in 2023. Reasons: unreliable results or conclusions; lack of ethics approval or compliance; concerns about the data; concerns about the peer review.

# Research on the Current Situation, Causes, and Countermeasures of Primary School Physical Education Teachers' Health Literacy

**DOI:** 10.1155/2022/7851028

**Published:** 2022-03-29

**Authors:** Lai Shangguan, Shu Chen, Lei Cao

**Affiliations:** Physical Education Institute, Hunan First Normal University, Changsha 410002, China

## Abstract

Under the background of healthy China, health education has been brought into the national education system. To improve the health literacy level of PE normal students in primary schools, this study studies the health literacy status of PE normal students in the “six-year junior middle school starting point system” using the methods of literature review, questionnaire survey, mathematical statistics, and so on. The results show that the health literacy level of “six-year junior high school starting point” PE normal students is close to that of national college students, but the health literacy is overall low. The success rate of health literacy of six-year physical education normal students from high to low is health skills, health knowledge, healthy lifestyle, and behavior; six-year physical education normal students have a high level of health skills, but a low level of healthy lifestyle and behavior. Countermeasures are put forward: optimizing the curriculum structure and strengthening health education; paying attention to health literacy and improving learning awareness; cultivating health awareness; maintaining the law of life, etc.

## 1. Introduction

As the country's largest primary school teacher education and public funds oriented rural primary school teacher training colleges, Hunan First Normal University took the lead in 2010 in the country to start the “starting point of junior high school six-year consistent system” primary education undergraduate professional training program. According to the mode of “starting point of junior middle school and six-year consistency; comprehensive training and directional development; integration of three natures and trinity; practice orientation and ability first,” we plan to recruit fresh excellent junior middle school graduates in rural areas to cultivate excellent primary school teachers. Based on this, the primary school physical education teachers of “six-year system from the beginning of junior high school” came into being. Health literacy refers to the individual's ability to access, understand, and process basic health information or services and make correct judgments and decisions to maintain and promote health and quality of life [1]. “2030 Planning Outline of a Healthy China” proposes to establish a school health education implementation mechanism focusing on primary and secondary schools. The generation of high-quality, high-level, and all-round students' health literacy has put forward higher requirements for physical education teacher education in the new era [2]. As early as the “Guidelines for Health Education in Primary and Secondary Schools” issued by the Ministry of Education in 2008, “Physical Education and Health” courses should be the main carrier of health education in primary and secondary schools at the grassroot level, and health education teachers should be based on the existing full-time and part-time health education teachers and physical education teachers. Therefore, it is necessary to pay attention to health for the reform and development of physical education teachers in China. Physical education teachers should know health, learn health, use health, and teach health [3].

The health literacy level of the “six-year system from the beginning of junior high school” primary school physical education normal students will directly affect the primary school students' health education and physical and mental health. Therefore, through the investigation and analysis of the health literacy status of six-year normal college students in Hunan First Normal University, including health knowledge, health skills, healthy lifestyle, and behavior, this study finds out the factors that restrict health literacy and puts forward some countermeasures to improve the health literacy level of normal college students.

“Health Literacy of Chinese Citizens-Basic Knowledge and Skills” was the first health literacy scale compiled by experts organized by the Ministry of Health of China in 2008 according to the national conditions of China. The scale was further improved and updated later. Taking the health literacy of the “six-year system sports normal students from the starting point of junior high school” in Hunan First Normal University as the research object, this study randomly selects 150 “six-year system sports normal students” from junior and senior high schools as the samples and selects some health knowledge points in “66 Articles on Health Literacy of Chinese Citizens” to evaluate the health literacy of the samples by means of questionnaire. According to the needs of research objectives and tasks, and based on Chinese Citizens' Health Literacy-Basic Knowledge and Skills, the Health Literacy Questionnaire for Physical Education Normal Students of “Six-year System at the Beginning of Junior High School” was designed. A total of 150 questionnaires were distributed, and 138 were recovered, with the recovery rate of 92%. The data of the questionnaires were analyzed, and the invalid questionnaires were cleared. The valid questionnaires were numbered, and the data were collated and analyzed.

## 2. The Current Situation of Health Literacy of Six-Year PE Normal School Students

### 2.1. The Overall Health Literacy Level of Six-Year PE Normal Students

School health education is the fundamental way to form citizens' health literacy [4].Physical education teachers' health literacy level plays a key role in school health education. For this purpose, we designed a questionnaire about the overall health literacy level of six-year normal college students majoring in physical education (Table 1). The title of the questionnaire came from Chinese Citizens' Health Literacy-Basic Knowledge and Skills. The three dimensions of the designed health literacy questionnaire included the following: health knowledge (12 questions), health skills (7 questions), and healthy lifestyle and behavior (10 questions), totaling 29 questions. The question type is single choice, and the answer to each question is correct, with 1 point; the answer to the question is wrong, with no score; and full scores are 29 points. According to the requirements of Health Literacy of Chinese Citizens-Basic Knowledge and Skills, the ones whose measurement scores in three dimensions accounted for more than or equal to 80% of their total scores were considered to meet the criteria. Therefore, based on the total score of 29 points, the overall health literacy achievement standard was 23.2 points (29 points ×80% = 23.2 points), of which 62 people reached the standard, with the achievement rate of 44.9%; similarly, the total score of health knowledge accomplishment was 12 points, with the judgment criterion of ≥9.6 points, and 67 subjects reached the standard, with the compliance rate of 48.6%; the total score of health skills was 7 points with the judgment standard of ≥5.6 points, and 70 subjects reached the standard, with the compliance rate of 50.7%; the total score of healthy lifestyle and behavior was 10 points, with the judgment standard of ≥8.0 points. There were 48 people who reached the standard, and the compliance rate was 34.8%.

From the statistical data, the overall success rate of health literacy of six-year normal university students is only 44.9%, which is not more than half of the total number surveyed. Moreover, the success rate of health literacy of six-year normal university students is ranked as health skills (50.7%), health knowledge (48.6%), and healthy lifestyle and behavior (34.8%) from high to low. In the three-dimensional health literacy of six-year PE normal students, only the average score of health skill level was 6 points, which exceeded the judgment standard (≥5.6), and the health knowledge, healthy lifestyle, and behavior were lower than the judgment standard, indicating that the health literacy of six-year PE normal students in health knowledge, healthy lifestyle, and behavior was not optimistic (Table 1).

The extensive health knowledge not only makes the six-year PE normal students handy in the school health education and teaching, but also can adjust themselves in time, using positive emotional contagion students. However, mastering strong health skills enables physical education teachers to calmly deal with unexpected events and deal with them in time to avoid accidents. At the same time, “learning high for the teacher, the body is for the model,” six-year physical education normal students' own healthy lifestyle and behavior habits are imperceptibly followed by students and have a greater impact on primary school students. However, the results of the survey show that the overall level of health literacy of six-year normal college students is on the low side. College is a crucial period for acquiring knowledge and forming various behavioral habits and lifestyles, as well as a golden period of health education. Health literacy acquired during this period can affect their current and adult health [5]. Therefore, it is necessary to strengthen the health education of PE normal students to improve their health literacy level.

### 2.2. The Success Rate of Health Literacy of Six-Year Normal Students in Different Categories

The first is in terms of gender. The comparison of health literacy among six-year PE normal school students from the perspective of gender (Table 2) reveals that there is no significant difference between male and female students. The overall success rates of health literacy for male and female students are 44.7% and 45.6%, respectively. The overall health literacy of female students is slightly higher than that of male students. From the three dimensions of health literacy, the rate of health knowledge reaching the standard was 43.5% for boys and 47.7% for girls; the success rate of health skills was 52.3% for boys and 51.6% for girls; the compliance rate of healthy lifestyle and behavior was 32.8% for boys and 35.1% for girls. Female students' literacy in the dimensions of health knowledge and healthy lifestyle was slightly higher than that of male students, which reflected that female students' health awareness was stronger than that of male students' health awareness, and they paid attention to their health habits and the relatively regular living schedule at ordinary times. On the contrary, in the dimension of health skills, boys are slightly higher than girls, which may be related to the relatively strong hands-on ability and adaptability of boys.

The second is in terms of age. The results of Table 2 show that the health literacy of six-year normal college students in different grades has no great difference on the whole. The overall success rate of health literacy is 45.3% in junior and 44.6% in senior. In the aspect of health knowledge, the rates of reaching the standard of junior and senior were 43.5% and 44.7%, respectively. In the aspect of health skill accomplishment, the junior and senior students have similarities, and the rate of reaching the standard is higher, 51.3% and 52.2%, respectively; in terms of healthy lifestyle and behavior, the compliance rates of junior and senior students are relatively low, 35.8% and 34.1%, respectively. Statistics show that the rate of reaching the standard of health knowledge of senior students is higher than that of junior students, but the number of reaching the standard has not yet exceeded half of the total number surveyed, indicating that the six-year normal college students do not have enough health knowledge after their studies in university. The compliance rate of the healthy lifestyle of junior high school students is higher than that of senior high school students, which is largely related to the more curriculum arrangement and more regular life of junior high school students. On the contrary, four senior students have relatively few courses and plenty of free time, neglecting their healthy lifestyle and behaviors, so the rate of reaching the target is low. Therefore, it is necessary to effectively strengthen the cultivation of a good lifestyle for senior PE normal students.

### 2.3. Three-Dimensional Health Literacy of Six-Year PE Normal Students

Health literacy is a synthesis of health knowledge and concepts, health skills, and healthy behavior, as well as physical, mental, and social health [6]. The first is health knowledge. A survey of health knowledge of six-year normal college students in physical education was conducted from 12 aspects, including healthy psychology, normal blood pressure values, normal body temperature of adults, normal pulse of adults, daily sleep time, transmission route of AIDS, nondiscrimination against patients, public health service, cockroach-transmissible diseases, the role of vaccination, early cancer signal, and fracture measures (Table 3). Judging from the health knowledge answering situation of six-year normal PE students, the scores on healthy psychology, AIDS transmission route, nondiscrimination against patients, and public health service are higher, 93.5%, 85.5%, 95.7%, and 89.9%, respectively. This indicates that the six-year normal PE students have a clear concept of physical and mental health and have a good grasp of AIDS transmission route. On the contrary, the methods for preventing the spread of animal diseases and cancer were insufficient, with the correct rates of 37.7% and 31.2%, respectively. As the future primary school physical education teachers, the lack of health knowledge of six-year physical education normal students will affect their work in primary school physical education and health education and teaching, so it is very important to strengthen their health knowledge learning.

The second is health skills. The survey was mainly conducted from seven indicators including emergency medical telephone number, definition of OTC, use of thermometer, measurement of pulse, identification of inflammable and explosive signs, rescue of electric shock, and fire alarm telephone number (Table 3). Statistical data show that, among the three dimensions of health literacy, the health skill literacy of six-year normal college students is the best, which has a high degree of similarity with the health literacy level of sports majors studied by scholars. This is related to the physical education major students' strong practical ability, quick and quick response, and generally able to calmly deal with dangerous situations. Among them, the awareness rates of “emergency medical emergency call” and “fire alarm call” were higher, 95.7% and 89.9%, respectively. It shows that the overall health skills of six-year PE normal students are relatively strong. Of course, health skills and health knowledge are complementary to each other, and health skills are based on certain health knowledge. Relatively speaking, the health medical skills of the six-year PE normal students are still relatively lacking. For example, the correct rates of “measuring pulse” and “rescuing the electric shock victim” are 68.1% and 60.9%, respectively. Therefore, physical education departments in colleges and universities should urge students to carry out systematic study and training of healthcare knowledge and skills, adhere to the combination of health theory knowledge and skill practice, and effectively improve the health skills of physical education normal students.

Finally, there are the aspects of healthy lifestyle and behavior. The survey was conducted with 10 indicators including meat and vegetable collocation, nutrition in diet, not sharing towels with others, health examination, frequency of toothbrushing, smoking and alcohol abuse, staying up late, use of antibiotics, treatment of animal scratch, and safe driving (Table 3). Statistics showed that healthy lifestyle and behavior were the ones with the lowest scores in the three dimensions of health literacy, especially “staying up late,” “healthy physical examination,” “diet and nutrition,” and “meat and vegetable collocation,” with the low correct rates of 16.7%, 28.3%, 42%, and 53.6%, respectively. This is related to the relatively free schedule of college students, who stay up very late. Among them, the majority of boys stay up late and drink heavily. At the same time, the six-year normal college students seldom take part in the physical examination and lack the consciousness of health examination, which reflects their low attention to body health. In addition, most of the students do not pay attention to food mix, do not like to eat vegetables, and have bad eating habits. Fortunately, we did a good job in brushing our teeth and driving safely, and the correct rates were 82.6% and 84.8%, respectively.

In conclusion, among the three dimensions of health literacy, the possession rate of health skills for six-year PE normal students is the highest, followed by health knowledge and finally the healthy lifestyle and behavior, and the score rate of different contents in each dimension is different. The health literacy level of college physical education teachers is improved, and then, their health status and teaching ability [7]areimproved. Therefore, the health education of six-year PE normal students should be targeted, focusing on strengthening their health knowledge and healthy lifestyle education, with a healthy lifestyle as the leading and with health knowledge as the auxiliary, and effectively improve the health literacy ability and level of six-year PE normal students.

## 3. Six-Year Physical Education Students' Health Literacy Constraints

### 3.1. Deficiency of School Health Curriculum

Modern curriculum theory believes that the curriculum pillar is the level of physical and mental development of the educated, the requirements and possibilities offered by future economic and social development, and the sum of knowledge, skills, and competencies involved in the curriculum [8]. From the point of view of the current physical education teacher education curriculum system, mainly to the physical education discipline education class curriculum, and health education class curriculum is missing, the current curriculum system is not conducive to the cultivation of physical education teachers' health education ability [9]. At the same time, the low level of basic knowledge and concept literacy to some extent reflects the marginalization and weakening of school health education [10]. Through the analysis of the training plan of six-year PE normal school students, we know that no health education-related courses have been found in the training courses. In addition, the survey on “the situation of setting up health education courses” for six-year PE normal students also revealed that students unanimously answered that no health courses were set up in schools, and even most students were not clear about which health education courses were specifically included. It shows that there is a lack of health education curriculum in the training curriculum system of six-year normal PE students. Students lack systematic study of health knowledge and skills, which results in the overall health literacy of six-year normal college students in physical education being not high.

### 3.2. Lack of Attention to Health Literacy

Health literacy comes from health education and is closely related to health behaviors. It has the characteristics of comprehensiveness, hierarchy, interaction, lifetime, and purpose [11]. In the survey of health knowledge learning habits of six-year PE normal students, 56 students (40.6%) took the initiative to learn, while 82 students (59.4%) did not take the initiative. Obviously, most of the six-year PE normal students do not pay enough attention to health knowledge, lack the consciousness of active learning, and have not formed the habit of learning health knowledge. Judging from the feedback of the answers to the health knowledge questionnaire, most of the six-year PE normal students have a vague and one-sided understanding of health knowledge, and even some conventional concepts have their understanding deviated. For example, for the understanding of health problems, 7% of students simply think that the so-called health refers to physical health and ignore the mental health.

### 3.3. Bad Lifestyle and Behaviors

Among the three dimensions of health literacy, the possession rate of healthy lifestyle and behavior of six-year PE normal students is the lowest, which indicates that they lack healthy lifestyle and behavior. Among them, staying up late existed and was serious for both boys and girls, with only 16.7% of them not staying up late, indicating that most students slept late at night and did not form good work and rest habits; on the issue of health check-up, only 28.3% of the students did the regular check-up, the rest of the students did not have the habit of physical examination; regarding “diet nutrition” and “meat and vegetable collocation” in daily life, the possession rates of six-year PE normal students are not high, 42.0% and 53.6%, respectively. It is well known that smoking and alcohol abuse does great harm to body. However, the survey shows that the rate of smoking and alcohol abuse is low (65.2%), and most of them are female students. Smoking and alcohol abuse among male students is especially serious. On the whole, the bad lifestyle has also become the bottleneck of the development of health literacy of six-year PE normal students.

## 4. Six-Year System of Sports Normal Students' Health Literacy Promotion Countermeasures

### 4.1. Optimize the Curriculum Structure and Strengthen Health Education

As the future primary school physical education teachers, the six-year system physical education normal students bear the responsibility and obligation of primary school physical education and health education. They should not only master solid sports professional knowledge and skills, but also have higher health literacy. Only in this way, we can meet the requirements of “healthy China” on school physical health education. However, compared with the sports knowledge and skills, the health literacy of six-year PE normal students is much lower. The reason is closely related to their lack of systematic study of health education curriculum. The content of health education is more directed to health knowledge, hygiene habits, lifestyle, environmental improvement, disease prevention, risk prevention, etc., which are less involved in the professional curriculum for physical education teacher training [12]. The survey also shows that the courses for six-year PE normal students are mainly cultural general knowledge courses and professional skill courses, and the health education courses to improve students' health literacy are in a state of deficiency. Therefore, the PE departments in colleges and universities should change the traditional PE teachers' educational concept and establish the talent cultivation concept of keeping pace with the times according to the requirements of “healthy China” on school health education. While focusing on the cultivation of sports professional skills, the structure of training courses is optimized and health education courses are reasonably added. For example, adding personalized health such as medical treatment, health care, fitness, and entertainment and field survival, to strengthen the health education of physical education normal students and improve the students' health education ability and level. In addition, it can actively expand low-cost, high-efficiency health education activities, for example, using the Internet, mobile phone text messages, and mobile phone WeChat.

### 4.2. Pay Attention to Health Literacy and Improve Learning Awareness

The six-year normal college students of PE are keen on learning PE professional skills and hold a dispensable attitude towards learning health knowledge and skills. For example, 59.4% of the students did not take the initiative to learn health knowledge. This awareness of not paying attention to health literacy is affected by social, school, and individual students and other factors, but the main reason is the lack of understanding of individual students. The acquisition of health knowledge and skills cannot be achieved overnight; it is a long process of accumulation. Therefore, sports normal students should attach great importance to their own health literacy acquisition, improve learning awareness, actively strengthen the study of health knowledge and skills, and effectively improve their own health education literacy.

### 4.3. Cultivate Health Consciousness and Keep the Law of Life

From the three dimensions of health literacy, the six-year PE normal students lack the most healthy lifestyle and behavior. The most prominent ones included staying up late, physical examination, diet and nutrition, and meat and vegetable dishes. Among them, staying up late was especially serious. Only 16.7% of the students did not stay up late. The reason for this is mainly due to the lack of health awareness among students. Therefore, it is essential to cultivate health awareness and a positive and optimistic attitude towards life. Only by establishing health awareness, they can actively resist junk food and avoid overeating, and even in the face of the temptation of endless food, they can self-control and then gradually form the habit of healthy eating. At the same time, with the gradual increase in health awareness, the phenomena of staying up late, smoking and drinking, and irregular life will also decrease sharply. Consciousness determines behavior. A healthy lifestyle is gradually formed, and life becomes more regular under the control of health consciousness.

## Figures and Tables

**Table 1:** Six-year normal college students' overall health literacy questionnaire (*n* = 138).

Health literacy	Question quantity *∗* score	Aggregate score	Criterion	Mean score	Number of people reaching the target	Compliance rate (%)
Overall health literacy	29 *∗* 1	29	≥23.2	20.6	62	44.9
Health knowledge	12 *∗* 1	10	≥9.6	8.1	67	48.6
Health skills	7 *∗* 1	7	≥5.6	6	70	50.7
Healthy lifestyle and behaviors	10 *∗* 1	10	≥8.0	6.3	48	34.8

**Table 2:** Attainment rate of health literacy of six-year normal college students in different categories.

Category		Overall health literacy (%)	Health knowledge (%)	Health skills (%)	Healthy lifestyle and behavior
Gender	Man	44.7	43.5	52.3	32.8%
	Woman	45.6	47.7	51.6	35.1%
Grade	Junior	45.3	43.5	51.3	35.8%
	Senior	44.6	44.7	52.2	34.1%

**Table 3:** Three-dimensional health literacy of six-year normal college students majoring in physical education (*n* = 138).

Health knowledge	Score number of people	Accuracy rate (%)	Health skills	Score number of people	Accuracy rate (%)	Healthy lifestyle and behaviors	Score number of people	Accuracy rate (%)
Health psychology	129	93.5	Medical emergency call	132	95.7	Meat and vegetable collocation	74	53.6
Blood pressure value	67	48.6	Fire alarm phone number	124	89.9	Dietary nutrition	58	42.0
Adult normal body temperature	96	69.6	Identify inflammable and explosive signs	119	86.2	Do not share towels	109	79.0
Adult normal pulse	65	47.1	Use a thermometer	106	76.8	Health check-up	39	28.3
Daily sleep time	93	67.4	OTC meaning	97	70.3	Number of times you brushed your teeth	114	82.6
Route of transmission of aids	118	85.5	Measuring pulse	94	68.1	Smoking and drinking	90	65.2
Nondiscrimination against patients	132	95.7	Rescue the electrocuted	84	60.9	Stay up late	23	16.7
Public health services	124	89.9				Antibiotic use	102	73.9
Cockroach-transmitted disease	52	37.7				Animal scratch treatment	98	71.0
The role of vaccination	103	74.6				Safe driving	117	84.8
Early signs of cancer	43	31.2						
Fracture measures	92	66.7						

## Data Availability

The datasets used and/or analyzed during this study are available from the corresponding author on reasonable request.
